The article "Modeling and Simulation in an Aircraft Safety Design Based on a Hybrid AHP and FCA Algorithm" was published in 2022. Journal: Comput Intell Neurosci.

# Modeling and Simulation in an Aircraft Safety Design Based on a Hybrid AHP and FCA Algorithm

**DOI:** 10.1155/2022/6424057

**Published:** 2022-05-27

**Authors:** Miaosen Wang, Yuan Xue, Kang Wang

**Affiliations:** Aeronautics Engineering College, Air Force Engineering University, Xi'an 710038, China

## Abstract

Throughout the world, the reliability-based approach to safety design of aircraft systems is quite mature and widely used. However, there are still shortcomings in the reliability-based aircraft system safety analysis method. It cannot dynamically analyze the accident evolution process and lack consideration of the complex situation of multifactor coupling. On the basis of the original aircraft system safety analysis method, this paper innovatively proposes a functional hazard analysis (FHA) method based on the analytic hierarchy process (AHP) and multifactor fuzzy comprehensive assessment (FCA). The purpose is to improve the objectivity and quantification of the FHA method in the safety design of aircraft systems. At the same time, in the terminal airworthiness verification, this paper proposes a repeatable and controllable virtual test flight verification method, which aims to reduce the cost and cycle of the terminal airworthiness verification and expand the coverage of the envelope verification. Finally, combined with the clauses in MIL-HDBK-516B, a case calculation is carried out to verify the feasibility of the proposed method.

## 1. Introduction

At present, the aircraft safety design can adopt either the reliability-based aircraft system safety design method [1–4] or the aircraft safety simulation design method based on modeling simulation [5–9]. Among them, the first method, aircraft system safety design, mainly aims at the safety of the aircraft itself and puts forward reliability design requirements for each system. The second method, aircraft safety simulation design based on modeling and simulation, can comprehensively consider the safety of aircraft from all aspects that affect the safety of aircraft operations. Based on the comprehensive system safety analysis method, the safety analysis of the aircraft itself is carried out, and the behavior characteristics of the man-machine-environment complex system are modeled and simulated, so as to realize the modeling, simulation and virtual design of the aircraft safety.

In the current environment, two methods of aircraft safety design are shown in Figure 1.

There are five potential application methods as shown in Figure 2: (1) FHA(function hazard analysis) based on virtual flight test and system safety evaluation; (2) PSSA(preliminary system safety analysis) security index assignment based on subjective and objective combination weighting; (3) SSA(system safety analysis) security based on virtual flight test as well as FTA(fault tree analysis) comprehensive verification and optimization of performance indicators; (4) airworthiness compliance verification based on virtual flight test; (5) the consideration of preventing multifactor accidents is added to CCA(canonical correlation analysis). All five of these potential applications are currently topical issues in aircraft safety design and deserve to be investigated.

This paper focuses on the exploratory research on Articles 1 and 4 (shaded parts). FHA based on virtual flight test and system safety evaluation (Section 3) and airworthiness compliance verification based on virtual flight test are investigated. (Section 4). The aim of this paper is to improve the process of aircraft system safety design and to innovatively investigate the functional hazard analysis method based on virtual flight test (VFT) and the functional hazard analysis method based on multifactor hierarchical analysis—fuzzy comprehensive assessment. For aircraft system safety design, most people still use fault-tree-based analysis, which cannot dynamically analyze the evolution of the accident process. The research method in this paper is a good way to study the evolution of accidents dynamically.

## 2. Related Work

Western countries have studied flight safety more extensively and meticulously and have conducted more in-depth research on the basic theory of flight safety, safety evaluation, and safety design. The US Army put forward safety systems engineering in the 1960s, with accidents as the main research subject, including safety analysis, safety measures and safety evaluation, and other major contents. The accident mechanism analysis models such as 'Heinrich's theory, accident chain theory, 'Murphy's theorem, SHEL model, and human-machine loop theory in system safety engineering have been widely used in flight safety research [10]. In particular, the international civil aviation community has incorporated human factors engineering and other theories to strengthen the study of “human-machine” and “human-loop” systems [11]. For example, research on cockpit resource management and reliability management began in the 1980s [12]. Baker, the University of Birmingham, UK, analyzed the impact of human factors and organizational behavior in aviation accidents [13]. Ramus of the University of California, USA, has also studied “human-loop” systems [14].

At present, developed countries in Europe and the United States have adopted the idea of system safety design methods [1–4] as the main approach in aircraft safety design, supplemented by methods based on virtual prototyping and virtual testing and evaluation of human-machine-loop complex systems [15–17]. The US military's fourth-generation warplanes, as well as aircraft design giants such as Boeing and Airbus that produce the B787 and A380, have undergone system safety design, and the safety design of European countries such as the UK, France, and Germany has basically referred to the US approach. At the same time, European and American countries have consistently attached importance to the simulation of aircraft functional hazards in the aircraft design and development phase, which has reduced design costs and shortened the design cycle, improved the intrinsic safety of the aircraft throughout its life cycle, and effectively reduced the probability of catastrophic accidents [17].

The simulation modeling method is also the mainstream method for studying engineering problems in the world today, whether it is the image tracking of UAVs [18–21] or on engine calibration and verification [21, 22]. There has been a lot of progress. In the field of aviation, simulation modeling is mainly used for the construction of dynamic models [23, 24] and so on.

Although the FHA method based on the analytic hierarchy process and multifactor fuzzy comprehensive assessment has many advantages, the fuzzy comprehensive assessment method is to comprehensively evaluate the influence of various influencing factors of a thing on the target in a fuzzy environment. The evaluation steps are as follows: first, establish the influencing factor set of the evaluation object; second, establish the target-based evaluation level and the weight set of each factor relative to the target; third, determine the membership degree of each factor; fourth, establish the fuzzy evaluation matrix. The fifth is to use fuzzy number sequence for comprehensive evaluation. The limitation of this method is that it is a complex work to establish the evaluation level of the target and the weight set of each factor relative to the target, which requires a lot of experience to find a suitable weight set. At the same time, a large amount of data are needed to verify whether the membership of each factor is accurate. The use of hierarchical analysis first requires the hierarchy of questions to derive a comparative judgement matrix for the next level relative to the previous level of factors based on subjective judgement, in which there is still an element of subjective judgement that may affect the accuracy of the weights in the later calculations.

## 3. Functional Hazard Analysis (FHA) Method Based on VFT and AHP-FCA

### 3.1. Research Ideas on Functional Hazard Analysis

The previous functional hazard analysis (FHA) is mostly analogy or evaluation based on experts' experience, which is highly subjective. The research methods proposed by FHA in this paper are mainly divided into the following two categories:

1. For thrust and control, flight control, etc., that can be studied through modeling, comprehensive research can be carried out by using the virtual flight test (VFT) and comprehensive fuzzy assessment (FCA).
2. Study on comprehensive fuzzy evaluation of functional hazards that are not easy to model, such as personnel life protection, comfortable environment for personnel (providing interior and living facilities, cargo compartment lighting, water supply, and drainage), special protection (fire prevention, firefighting, anti-icing, de-icing), and other functional hazards (FCA) methods for research.

### 3.2. Case Analysis of the Functional Hazard Analysis Method in a Virtual Flight Test

The following is a case study of simulation analysis of the system. Set a certain type of aircraft with dual engines, as well as model and simulate the functional hazard of “thrust loss of single engine, resulting in a serious thrust asymmetry,” which mainly causes the reduction of thrust and yaw moment. The impact model of a single engine is established, and the functional hazard impact model of unilateral engine failure is added to the virtual flight test safety analysis system for simulation. The simulation visual map is shown in Figure 3.

According to the simulation analysis, the main risk after a single engine shutdown is the final landing stage. Considering only the risk caused by a single engine failure, the following three types of accidents may occur:

1. The runway is misaligned, and the landing gear is broken off the runway, causing fire or damage to the aircraft structure. The critical safety parameter is the dangerous landing distance, as shown in Figure 3(c).
2. The descent rate is too large, and the landing gear is broken on the runway, causing fire or damage to the aircraft structure. The decisive parameter of safety is the descent rate at the moment of touchdown, as shown in Figure 3(d).
3. During the landing phase, the flight gets out of control in the air and crashes outside the runway. The decisive safety parameter is the angle of attack or sideslip, as shown in Figure 3(e). The three-dimensional graphs of various situations are shown in. After 300 virtual flight test simulations, the proportions of the above three types of accidents after a single engine failure are 15.3%, 22.1%, and 10.5%, respectively. To sum up, the major accidents that indicate the danger of this function may lead to the destruction of the aircraft are classified as a disaster (Class I) [3], which is consistent with the actual situation.

### 3.3. FHA Based on Improved AHP-Fuzzy Comprehensive Assessment (AHP-FCA)

At present, the database data used for system safety analysis in China are not comprehensive, as shown in Figure 4, so it is difficult to establish mathematical models for some FHA projects, such as personnel life protection, personnel comfortable environment (providing interior decoration and living facilities, cargo compartment lighting, water supply and drainage), and special factor protection (fire prevention, fire extinguishing, anti-icing, deicing, etc.). Fuzzy comprehensive assessment (FCA) can control the influence of the subjective factors of evaluation information on the evaluation results to a smaller extent, making the evaluation more comprehensive and objective. It is suitable for multisubjects to multilevel and multicategory indicators. In recent years, the advantages of evaluation information integration have been rapidly developed and widely used [25, 26]. Therefore, this paper proposes a method of applying fuzzy comprehensive assessment (FCA) to evaluate some functional hazard analysis items that are difficult to model.

In this paper, the fuzzy comprehensive evaluation and analytic hierarchy process methods are organically combined and introduced into the qualitative analysis of FHA, and the FHA method of multifactor fuzzy comprehensive evaluation based on the analytic hierarchy process is proposed. The general steps of the method are shown in Figure 5.

### 3.4. Improved AHP-Fuzzy

#### 3.4.1. Comprehensive Evaluation Method

For the evaluation of complex issues, there are many factors that need to be considered, and these factors may also belong to different levels. Therefore, all factors can be divided into several categories according to certain attributes, and the first category can be carried out in each category. The first-level comprehensive evaluation and the second-level comprehensive evaluation based on the results of various evaluations, and so on. The specific working steps are as follows:

(1) Let the evaluation set be *V*={*v*_1_, *v*_2_,…, *v*_*n*_}; For the domain of factors *U*, first divide it into *S* disjoint subsets according to the attributes of each factor; Assume each subset *U*_*k*_={*u*_*k*1_, *u*_*k*2_,…, *u*_*km*_}(*k*=1,2,…, *S*); For different subsets, the number of elements (*m*) can be different.
(2) According to the effect of each factor in the subset *U*_*k*_, the weight distribution of each factor is given. Different experts have different identifications of weights, and the constructed AHP matrix is different. In order to synthesize the opinions of multiple experts, this paper adopts the method of combining quantitative expert survey and AHP to determine the weight of evaluation factors. For a certain level of indicators:
  (a) Each expert constructs a judgement matrix for different factors *A*_*k*_, (*k*=1,2,…, *S*) and calculates the preliminary weight of each subitem indicator through the judgement matrix given by different experts; Experts also explain the familiarity with a certain indicator *r*, in which *r*=1 indicates that the expert is familiar with the content being evaluated; *r*=2 indicates that the expert is better familiar with the content being evaluated; and *r*=3 means that the expert is not familiar with the content being evaluated.
  (b) Assume that the weight of the *i* expert to the *j* index according to the importance of the factors is *a*_*ij*_, *y*_*ir*_ is the confidence weight of the *i* expert, and set *y*_*i*1_=1,  *y*_*i*2_=0.8,  *y*_*i*3_=0.5, where *i*=1,2,…, *n* is the total number of experts; *j*=1,2,…, *m* is the total number of indicators. Then, the comprehensive score of the index *j* is as follows:
    (1) $$\begin{array}{c} \bar{a_{j}}=\sum_{i=1}^{n}a_{ij}\frac{y_{ir}}{\sum_{i=1}^{n}y_{ir}},\;i=1,2,\ldots ,n,\;j=1,2,\ldots ,m. \end{array}$$
  (c) The normalization of index weight is as follows:
    (2) $$\begin{array}{c} a_{j}=\frac{\bar{a_{j}}}{\sum_{j=1}^{m}\bar{a_{j}}},\;j=1,2,\ldots ,m. \end{array}$$
  Similar to the above method, the weights of other indexes of each layer can be obtained, and the weights of each layer are set as follows:
    (3) $$\begin{array}{c} a_{k}=\left[a_{k1},a_{k2},\ldots ,a_{km}\right]\left(k=1,2,\ldots ,S\right)\sum_{j=1}^{m}a_{kj}=1. \end{array}$$
(3) Comprehensive evaluation is carried out within the scope of each factor subset *U*_*k*_, and the fuzzy evaluation matrix **r**_**ki**_=(*i*=1,2,…, *m*) composed of fuzzy vectors is obtained **R**_**k**_, namely,
  (4) $$\begin{array}{c} R_{k}=\left[\begin{array}{c} r_{k1}\\ r_{k2}\\ \vdots \\ r_{km} \end{array}\right]=\left[\begin{array}{cccc} r_{k11} & r_{12} & \cdots & r_{k1n}\\ r_{k21} & r_{k22} & \cdots & r_{k2n}\\ \vdots & \vdots & \vdots & \vdots \\ r_{km1} & r_{km2} & \cdots & r_{kmn} \end{array}\right]\left(k=1,2,\ldots ,S\right). \end{array}$$
Then, calculate the corresponding evaluation grade membership vector *b*_**k**_ according to formula (5), namely,
  (5) $$\begin{array}{c} b_{k}=a_{k}oR_{k}=\left[b_{k1},b_{k2},\ldots ,b_{kn}\right]\left(k=1,2,\ldots ,S\right). \end{array}$$
(4) Let **a** be the factor-action fuzzy vector of *S* subsets of factors, and its expression is **a**=[*a*_1_, *a*_2_,…, *a*_*S*_] , where *a* is the weight distribution of the importance of each subset, and is determined by improved AHP. Then, the mathematical formula of the second-level fuzzy evaluation is **b**=[*b*_1_, *b*_2_,…, *b*_*n*_]=**a**∘**R**.Make a comprehensive judgement based on the results of *b.*

### 3.5. Multifactor Comprehensive Evaluation Application Case Calculation

According to the definition of functional hazard analysis in SAE ARP4761, the FHA fuzzy comprehensive evaluation system is established (Figure 6).

The evaluation is carried out according to the functional risk evaluation index system. Since each index cannot be evaluated by simple quantitative analysis methods, the multi-factor fuzzy comprehensive evaluation method is used to make fuzzy comprehensive evaluation of risks. The index system is divided into two layers, and two fuzzy methods are required for calculation.

According to the improved fuzzy comprehensive evaluation method, a civil aviation aircraft's “yaw damping function loss” is taken as an example to carry out functional hazard analysis, and the evaluation is based on the opinions of 10 experts.

The specific calculation process is as follows:

(1) Setting of the risk index system. The first-level indicators are divided into three categories: crew, passenger, and aircraft. The crew is divided into two categories that cause physical unsuitability and increase the workload. The passenger mainly causes physical discomfort. The aircraft is divided into two categories: reduced function (loss) and reduced safety margin.
(2) Classification of risk levels. According to the risk level in ARP4761, there are 5 levels can be formed: none (V), minor (IV), major (III), severe (II), disaster (I), and the abovementioned 5 evaluation level elements constitute a set of evaluation grades, that is *V* = (*none, minor, larger, serious, disaster*).
(3) Use the expert survey method and AHP method to determine the weight of evaluation factors, which are crew *a*_1_=0.4, passengers *a*_2_=0.4, and aircraft *a*_3_=0.2; *a*_11_=0.4,  *a*_12_=0.6,  *a*_21_=1,  *a*_31_=0.4,  *a*_32_=0.6
(4) Evaluate specific indicators:
  (6) $$\begin{array}{c} R_{1}=\left[\begin{array}{ccccc} 0 & 0.5 & 0.4 & 0.1 & 0\\ 0 & 0.2 & 0.6 & 0.2 & 0 \end{array}\right],\\ R_{2}=\left[\begin{array}{ccccc} 0.1 & 0.4 & 0.4 & 0.1 & 0 \end{array}\right],\\ R_{3}=\left[\begin{array}{ccccc} 0 & 0.3 & 0.6 & 0.1 & 0\\ 0 & 0.4 & 0.5 & 0.1 & 0 \end{array}\right]. \end{array}$$

The comprehensive evaluation is carried out according to the model *M*(•，+), then,

(7) $$\begin{array}{c} b_{1}=a_{1}\circ R_{1}=\left[\begin{array}{cc} 0.4 & 0.6 \end{array}\right]\circ \left[\begin{array}{ccccc} 0 & 0.5 & 0.4 & 0.1 & 0\\ 0 & 0.2 & 0.6 & 0.2 & 0 \end{array}\right]=\left[\begin{array}{ccccc} 0 & 0.32 & 0.52 & 0.16 & 0 \end{array}\right],\\ b_{2}=a_{2}\circ R_{2}=\left[1\right]\circ \left[\begin{array}{ccccc} 0.1 & 0.4 & 0.4 & 0.1 & 0 \end{array}\right]=\left[\begin{array}{ccccc} 0.1 & 0.4 & 0.4 & 0.1 & 0 \end{array}\right],\\ b_{3}=a_{3}\circ R_{3}=\left[\begin{array}{cc} 0.4 & 0.6 \end{array}\right]\circ \left[\begin{array}{ccccc} 0 & 0.3 & 0.6 & 0.1 & 0\\ 0 & 0.4 & 0.5 & 0.1 & 0 \end{array}\right]=\left[\begin{array}{ccccc} 0 & 0.36 & 0.54 & 0.1 & 0 \end{array}\right],\\ b=a\circ R=\left[\begin{array}{ccc} 0.4 & 0.4 & 0.2 \end{array}\right]\circ \left[\begin{array}{ccccc} 0 & 0.32 & 0.52 & 0.16 & 0\\ 0.1 & 0.4 & 0.4 & 0.1 & 0\\ 0 & 0.36 & 0.54 & 0.1 & 0 \end{array}\right]=\left[\begin{array}{ccccc} 0.04 & 0.36 & 0.48 & 0.12 & 0 \end{array}\right]. \end{array}$$

As the maximum degree of membership in *b* is *b*_3_=0.48, according to the principle of maximum degree of membership, the functional hazard is taken as greater (III), and the evaluation result is consistent with the actual situation corresponding to this type of aircraft.

In today's increasingly important flight safety, the functional hazard analysis method based on multifactor analytic hierarchy process-fuzzy comprehensive assessment has a good application prospect for aircraft safety. At present, the aircraft safety of major airlines mainly depends on the preflight inspection of the flight crew and the planned maintenance of the aircraft. Carrying out the preflight inspection according to the method proposed in this paper is helpful to the work of the flight crew and the improvement of the safety of the aircraft.

## 4. Airworthiness Compliance Verification Method Based on the Virtual Flight Test of a Complex System

“Aircraft Verification” is located at the end of the “V”-shaped diagram of the system safety design, which is mainly used to verify whether the aircraft meets safety requirements.

The verification method based on the virtual flight test of the complex system has the advantages of saving money, shortening cycle, good safety, and controllability. This paper focuses on the safety verification technology based on virtual flight test and conducts a case study in conjunction with the specific clauses in MIL-HDBK-516B [2].

### 4.1. Idea of Airworthiness Compliance Verification Based on the Virtual Flight Test

Aviation compliance verification methods usually include the following 10 types: declaration of conformity, documentation, calculation/analysis, safety evaluation, laboratory experiments, ground tests, flight tests, aircraft-level inspections, and equipment qualification inspections. In the verification of flight safety, the traditional methods of flight test and manual simulation have the following shortcomings [21]: The use cost of flight test is expensive, and the preparation as well as implementation cycle is long; it is difficult to exhaust all the driving in flight test and manual simulator [27–29]. Fields, especially in-flight restrictions involving complex boundary conditions; traditional T&E (Test and Evaluation) involves redesign and iteration of planning. Virtual flight test and evaluation (VT&E or VT&C) as a new flight test verification technology has great advantages [7]: First, it can conduct safety assessments on complex boundary states that cannot be carried out in flight tests to ensure the safety of the aircraft. Second, adding the virtual flight test in the design stage can shorten the design cycle and obtain more information about the airworthiness/safety of the aircraft. How to establish a reliable “pilot-aircraft-control environment” model, and use the effective simulation data to quantitatively evaluate and verify the airworthiness status is an urgent problem that needs to be studied [30–32].

The proposed airworthiness compliance verification method based on virtual flight test of complex system is shown in Figure 7. The pilot, aircraft, and operating environment are studied as a system, and the pilot-aircraft-operating environment model is established. Starting from FAR, JAR, АП, and other airworthiness standards, the flight test scenario library is obtained, and the pilot-aircraft operating environment is established.

The model realizes the virtual flight test, obtains the extreme value samples of decisive parameters, evaluates flight risk probability by applying flight safety quantitative evaluation theory, and proposes comprehensive evaluation conclusions and safety design improvement measures. The corresponding man-machine environment model and complex system model should be selected according to the establishment of the subject scenario database.

### 4.2. Establishment of a Database of Airworthiness Verification Subjects

The establishment of the scenario database is based on the analysis of the airworthiness clauses. Airworthiness standards are the basis of aircraft airworthiness verification. American civil aviation has relatively complete airworthiness standards, such as FAR 23, 25, 27, etc., in which there are specific regulations on the airworthiness requirements that the aircraft including its various systems, need to meet. CCAR series of Chinese civil aviation airworthiness standards are formed on the basis of American civil aviation standards. At present, the U.S. military has conducted airworthiness reviews on advanced fighters such as F-22 and F-35. The foundation is MIL-HDBK-516B, which sets detailed requirements for the aircraft systems. The first step of airworthiness review is to start with airworthiness standards and obtain airworthiness scenario database (equivalent to flight test risk subjects) according to the terms that need to be verified.

Disadvantages are the starting point of flight accidents. Therefore, the analysis of potential unfavorable factors based on the airworthiness verification clause is the basis of the establishment of the airworthiness scenario database. The analysis methods of unfavorable factors include failure mode and impact analysis (FMEA), event tree (ETA), fault tree (ETA), checklist method, engineering experience method, etc. In this paper, the module table is proposed to build the scene library. The basic function of the scenario library is to describe the possible accident chains in the verification of specific airworthiness clauses, which mainly includes potential unfavorable factors affecting flight safety, adverse effects on aircraft movement, and parameters that play a decisive role in flight safety. Taking Clause 6.2.4.2 of Chapter VI Flight Control Function (VCF) of MIL-HDBK-516B as an example, the process of establishing flight scenes is explained.

To apply the “barrel principle,” it is need to first find the weakest link of the fly-by-wire control system, that is, the link with a higher failure rate and a greater impact on flight safety. According to the flight record data and reliability test of this type of aircraft, the overload sensor and angular velocity sensor are the most vulnerable components.

Therefore, there are two potential accident chains caused by sensor failure. The failure of these two types of sensors led to the failure of elevator and aileron, respectively. Through simulation, the safety decisive parameter of the two accident chains is the angle of attack *α*, overload *n*_*z*_ or rolling angular velocity *p*. The scenario of this clause is shown in Figure 8.

According to the reliability experiment of a fly-by-wire control system, and the statistics of flight records of this type of aircraft, the components with the highest failure rate in the system are overload sensors and the roll angular velocity sensors.

### 4.3. Modeling and Simulation of Complex Situations

Establish the impact model of two types of equipment failures. The failure of the overload sensor of fly-by-wire control system may cause noncommand step deflection of the elevator, which may lead to noncommand pitching of the aircraft, resulting in the normal overload *n*_*z*_ and the distance change of the angle of attack *α* or even exceeding the limit. A negative tail deflection angle causes the aircraft to pitch up, which is more likely to cause stalls, and positive tail deflection angles are more likely to cause overload. Therefore, the decisive parameters of flight risk caused by positive and negative tail deflection angles are different. The failure mode model of the overload sensor is the stuck model:

(8) $$\begin{array}{c} y_{i\text{out}}\left(t\right)=a_{i}. \end{array}$$

According to the literature [13], the fault deflection value of the elevator deflection angle obeys the truncated normal distribution of the maximum and minimum values, and its value range is (−8deg, 8deg). The rolling angular velocity sensor obeys uniform distribution, and the mathematical expression of its fault model is as follows:

(9) $$\begin{array}{c} x_{i}=\left\{\begin{array}{cc} x_{it}, & \text{normal,}\\ x_{\text{min}}+\left(x_{\max}-x_{\min}\right)\times \text{Rand}\left(0,1\right), & \text{failure,} \end{array}\right. \end{array}$$

where *x*_*i*_ is the sensor display value, *R*, (0,1) is a (0,1) random number, and the upper and lower limit of the failure angle of aileron deflection is *x*_max_ and *x*_min_, respectively. The histogram of the failure angle of the elevator and aileron is shown in Figure 9.

The aircraft six-degree-of-freedom nonlinear differential equations are established in MATLAB. Based on the established pilot, aircraft model, and fault model, a virtual flight test system is established on the basis of MATLAB/SIMULINK and *FlightGear*. The failure angle and the driver's response after the failure are the inputs of the system simulation, and the outputs are the angles of attack, overload, and roll angular velocity. The flight of the two types of sensors after failure is simulated, and some of the simulation results are shown in Figures 10 and 11.

### 4.4. Airworthiness Compliance Verification and Analysis Conclusions

Based on Monte Carlo simulation of the complex system, extreme samples of angle of attack, overload, and roll velocity are obtained.

#### 4.4.1. Airworthiness Compliance Verification of Clause 6.2.4.2

*(1) Flight Risk Caused by Sensor Overload.* Based on the Monte Carlo method, 500 simulations are carried out, and 500 elevator failure deflection angles are obtained.

The probability of positive and negative declination is the same. The negative deflection angle causes the aircraft to pitch up sharply, whose safety decisive parameter is the angle of attack. Based on the RAE-PSO optimized generalized extreme value distribution model evaluation, the risk probability is obtained as *r*_1_=0.0468. The relationship between extreme value samples and standard deviation is shown in Figure 12.

Similarly, the flight risk caused by the negative deflection angle can be calculated. The decisive parameter is the negative overload, and the risk probability is evaluated as *r*_2_=0.0322, so *R*_1_=0.5 × (*r*_1_+*r*_2_)=0.0395.

The failure rate distribution of overload sensors obeys the Weibull distribution. Assume that when the subject is flying, the service time of the sensor system is 200 hours, and the failure rate is *λ*_1_=3.0 × 10^−6^/h, so the risk probability caused by the overload sensor failure is *Q*_1_=1/2(*r*_1_+*r*_2_)*λ*_1_=1.4 × 10^−6^/h. Meet the requirements of GJB2878-97.

*(2) Flight Risk Caused by the Failure of the Rolling Angular Velocity Sensor.* The maximum allowable rolling angular velocity of this type of aircraft is 90°/s. Based on the RAE-PSO optimized generalized extreme value distribution model, the estimated risk probability is *R*_2_=0.0683. The failure rate prediction model of the rolling angular velocity sensor obeys the exponential distribution model, and the failure rate is *λ*_2_=1.2 × 10^−5^. The risk probability per flight hour is: *Q*_2_=8.2 × 10^−7^/h, which does not meet the requirements of GJB2878-97.

#### 4.4.2. Airworthiness Compliance Verification of Clause 6.2.4.3

“Verify that the unfavorable factors affecting the control and structure of the fly-by-wire control system will not cause safety hazards to the aircraft and members in a short period of time.” This topic needs to verify the risk of telex control system under the influence of two unfavorable factors. This subject needs to verify the risk of the telex control system under the influence of two unfavorable factors. The failure rate of the overload sensor and rolling angular velocity sensor takes into account the influence of redundancy design. Sensor failure in flight cannot be repaired. The following multifactor situation tree model can be established (Figure 13).

(10) $$\begin{array}{c} \left\{\begin{array}{c} Q_{12}=\lambda_{1}R_{1}+\lambda_{1}S_{1}\lambda_{2}R_{12},\\ Q_{21}=\lambda_{2}R_{2}+\lambda_{2}S_{2}\lambda_{1}R_{21}. \end{array}\right) \end{array}$$

Since the two unfavorable factors are independent, the order can be regarded as random equal. *η*_12_ and *η*_21_ each takes 0.5, among which the single-factor situation risk probability. *R*_1_ and *R*_2_ has been calculated in the risk assessment above. Furthermore, *R*_12_ and *R*_21_ involve the simulation of the two-factor coupling situation. The faults of the overload sensor and rolling angular velocity sensor are simulated, respectively, which belong to the category of high-frequency events, and the Monte Carlo method is used for simulation evaluation. Set *R*_12_=0.35 and *R*_21_=0.43; then, the comprehensive risk probability is calculated as follows: *Q*=*η*_12_*Q*_12_+*η*_21_*Q*_21_=4.7 × 10^−7^/h, which meet the requirements of GJB2878-97.

It can be seen from the above cases that VT&E can perform safety assessment on the complex boundary states that cannot be carried out during the test flight process and has a non-negligible effect on the safety of the aircraft. If the virtual test flight evaluation is carried out on the aircraft in the design stage, more airworthiness data of the aircraft can be obtained, which has a good effect on the design of civil aircraft and military aircraft.

Flight risk is closely related to component failure rate and its role in the system. Therefore, the following three suggestions are put forward: (1) improve the reliability of overload sensors or replace them as soon as possible and (2) weaken the correlation between component failures and risks and improve the robustness of human-machine systems.

#### 4.4.3. Carrying Out Targeted Training for Drivers with Similar Failures

This method is applicable to the airworthiness verification of military and civilian aircraft, with the advantages of low cost, excellent repeatability, and controllability. It can be used as an effective supplement or substitute for the airworthiness verification method of complex high-risk flight test verification subjects. More comprehensive flight safety analysis data can be obtained within the whole flight envelope.

## 5. Conclusions

This paper studies the application method of modeling and simulation method in system security design. An improved aircraft system safety design process is proposed, and the functional hazard analysis method based on the virtual flight test (VFT) and the functional hazard analysis method based on multifactor AHP-fuzzy comprehensive assessment are studied. The airworthiness verification idea based on virtual test flight of the complex system is proposed. Combined with the Clauses in MIL-HDBK-516B, case calculations are carried out to verify the feasibility of the proposed method. However, the modeling and simulation and quantitative risk assessment of multifactor complex situations are heavy and difficult tasks. At present, there are not many achievements in China's quantitative research on the safety of multifactor and complex flight situations, coupled with the limited level of my own, the relevant research needs to be further improved and deepened. The follow-up research can be carried out from the following aspects:

1. Further improve the multifactor human-machine-loop and unfavorable factor model library.
2. Limited by time, energy, and other factors, the text only establishes models of some typical key systems and unfavorable factor models. There are many kinds of equipment failures, human-induced failures, and harsh environments, especially the human model is relatively abstract, and it is difficult to obtain data on the psychological and physiological characteristics of people under multifactor conditions. Therefore, the next step needs to further supplement and improve the models of key systems, equipment failures, and human errors.
3. Further strengthen the integration of modeling and simulation with the safety design process of aircraft systems.
4. The reliability-based system safety analysis method is mainly based on fault tree (FTA) analysis, which cannot dynamically analyze the accident evolution process. Into the research, the two have great differences in the overall thinking and specific modeling methods. This paper is only a preliminary exploratory study, and further research is required.
5. Strengthen the verification research on model verification and evaluation methods.
6. The final application of modeling and simulation depends on its true reliability. The next step should be to strengthen the VVA check of the modeling and simulation of multifactor complex systems. The proposed safety evaluation method and safety design method are also in the stage of preliminary application, and the proposed evaluation method should be further tested in practice in order to provide objective and effective theoretical support for flight safety in complex flight situations.

## Figures and Tables

**Figure 1:** Aircraft safety design methods.

**Figure 2:** Improved “V”-shaped program for safety design of the aircraft system.

**Figure 3:** Simulation view.

**Figure 4:** 3D simulation curve.

**Figure 5:** General steps of FHA based on AHP-FCA.

**Figure 6:** Schematic diagram of the FHA indicator system.

**Figure 7:** Airworthiness compliance verification idea map.

**Figure 8:** Accident chain scenario of Clause 6.2.4.2 in MIL-HDBK-516B.

**Figure 9:** Noncommand deflection of the elevator and aileron caused by two types of sensor failures.

**Figure 10:** Different perspectives in FlightGear.

**Figure 11:** Changes in the angle of attack, pitch angle, and pitch angle velocity caused by the sensor over time.

**Figure 12:** Relationship between extreme angle of attack and standard deviation.

**Figure 13:** Multifactor situation tree model. (a) Possible order 1. (b) Possible order 2.

## Data Availability

The data used to support the findings of this study are available from the corresponding author upon request.
